The article "Research on Optimization Scheme for Blocking Artifacts after Patch-Based Medical Image Reconstruction" was published in 2022. Journal: Comput Math Methods Med.

# Research on Optimization Scheme for Blocking Artifacts after Patch-Based Medical Image Reconstruction

**DOI:** 10.1155/2022/2177159

**Published:** 2022-07-31

**Authors:** Yan Xu, Shunbo Hu, Yuyue Du

**Affiliations:** ^1^College of Computer Science and Engineering, Shandong University of Science and Technology, Qingdao 266590, China; ^2^College of Information Science and Engineering Linyi University, Shandong Province 276005, China

## Abstract

Due to limitations of computer resources, when utilizing a neural network to process an image with a high resolution, the typical processing approach is to slice the original image. However, because of the influence of zero-padding in the edge component during the convolution process, the central part of the patch often has more accurate feature information than the edge part, resulting in image blocking artifacts after patch stitching. We studied this problem in this paper and proposed a fusion method that assigns a weight to each pixel in a patch using a truncated Gaussian function as the weighting function. In this method, we used the weighting function to transform the Euclidean-distance between a point in the overlapping part and the central point of the patch where the point was located into a weight coefficient. With increasing distance, the value of the weight coefficient decreased. Finally, the reconstructed image was obtained by weighting. We employed the bias correction model to evaluate our method on the simulated database BrainWeb and the real dataset HCP (Human Connectome Project). The results show that the proposed method is capable of effectively removing blocking artifacts and obtaining a smoother bias field. To verify the effectiveness of our algorithm, we employed a denoising model to test it on the IXI-Guys human dataset. Qualitative and quantitative evaluations of both models show that the fusion method proposed in this paper can effectively remove blocking artifacts and demonstrates superior performance compared to five commonly available and state-of-the-art fusion methods.

## 1. Introduction

In recent years, with the development of deep learning, medical imaging has gradually become one of the most promising fields of artificial intelligence. Especially in the aspects of localization and detection, recognition and classification, lesion segmentation, registration, and fusion in medical images, deep learning algorithms have played a crucial role in assisting doctors to diagnose accurately and efficiently [1]. Medical images have the characteristics of large image pixels [2], when using neural networks to process them, due to the limitations of computer video cards and video memory, directly using the original image as an input will often lead to insufficient graphics memory. The usual processing method involves slicing the original image, reconstructing the image patches, and then splicing the image patches. In deep learning, patch-based training methods have been widely used because they can save GPU memory, are not affected by insufficient training data, and can obtain better local performance than other methods [3]. However, there is also a grid artifact phenomenon at the edge of patches when they are spliced for image reconstruction as shown in Figure 1 [3], these artifacts are called image blocking artifacts.

To solve this problem, Yang et al. [4] and Hu et al. [5] obtained the final predicted deformation field by averaging the overlapping regions of patches when reconstructing the deformation field in medical image registration. In brain image registration using dual-supervised fully convolutional networks, as proposed by Fan et al. [6], only the deformation field in the central region of the patch is estimated, the input patch size is 64 × 64 × 64, and the output DDF (dense displacement field) is 24 × 24 × 24. The MINScnn model proposed by Müller and Kramer [7] used the average fusion method for the two overlapping patches in the segmentation field. In the patchify method proposed by Wu, the overlapping region is covered with the next patch [8]. The EDW (Exponential-Distance-Weighted) method proposed by Wu et al. [9] uses an exponential function to convert the distance between the point of the overlapping area and the center point of the patch into a weight coefficient and reconstruct the predicted deformation field by weighting. This method achieved good results.

During image reconstruction, most of the above methods reduce image blocking artifacts to a certain extent by reducing the step size or by performing estimates for the central area of the patch, but blocking artifacts are still obvious after image reconstruction. Considering the uncertainty of patch edge region prediction, we propose to use the truncated Gaussian function as a weighting function to convert the Euclidean distance from the points in the overlapping regions to the center point of the patch into a weight coefficient. The value of the weight coefficient will decrease with increasing distance, reducing the predicted value in the patch edge region. Finally, the reconstructed image will be obtained by weighted fusion. For distance calculation, we choose Euclidean distance as the distance measure [9]. This method can be applied to any patch-based deep learning network without modifying the network structure and loss function. Compared with the image reconstruction methods used in the above literature, the patch-based fusion method in this paper shows better performance in both qualitative and quantitative evaluations.

The paper is organized as follows. In Section 2, we briefly review the popularly available methods for extracting patches in deep learning.  Section 3 describes the proposed patch fusion method in detail. In Section 4, we evaluate the proposed patch fusion algorithm on synthetic and real datasets and present the experimental results. At the same time, a comparison with other state-of-the-art methods is also given. Conclusions and future works are discussed in Section 5.

## 2. Common Methods for Extracting Patches

Nonoverlapping slicing is performed directly on the image, as shown in Figure 2(a). Assuming that the image size is 512 × 512, the image is sliced into four equal parts, and the size of each patch is 256 × 256. The patches are input to the network to obtain the reconstructed image patches, and then, they are stitched together. Because the boundary information of each patch is inconsistent after reconstruction, the stitched image has obvious blocking artifacts.

In overlapping slicing, the image is sliced into patches, so that there are overlapping areas between the patches, as shown in Figure 2(b). The red region is the region where the two patches overlap. Assuming that the image size is still 512 × 512 and the red overlapping region is 8 pixels wide, then the size of the input patch is 260 × 260. After reconstruction, in situ pixel stitching is performed, and the red overlapping part is taken as the average value after stitching. This scheme has a better effect in removing the blocking artifact. However, since the average weighting method is adopted for the overlapping region, the weight of the pixels in the overlapping region is the same no matter how far away from the center point, so grid artifacts appear.

When padding is used around the image block, a patch is obtained as shown in block 1 in Figure 2(c). First, the padding is made around the image, the image is sliced after padding, and the cyan line is the central axis of the image. For example, in block 1, the orange part is the size of the original image block, and the surrounding red area consists of the expanded pixels. If the original image block is 256 × 256 and the red area occupies a width of 8 pixels, the input patch size is 272 × 272 (256 + 8∗2) for reconstruction. Then, the reconstructed image block is cut with a width of 8 pixels around to obtain a patch with a size of 256 × 256, and finally, it is stitched in sequence. For image block 1, the red part is removed after reconstruction. For image block 2, the blue part on the left needs to be cut off. This scheme is better than the previous two schemes in removing blocking artifacts, but it will be affected by stride. The smaller the stride is, the better the effect of removing blocking artifacts. However, the smaller stride, the greater the amount of calculations. Since the weight of the entire estimated central region is the same, the image blocking artifacts will still occur.

## 3. Methods and Theories

### 3.1. One-Dimensional Gaussian Distribution

The one-dimensional Gaussian function has the following form [10]:

(1) $$\begin{array}{c} f\left(x\right)={ae}^{-{\left(x-b\right)}^{2}/2c^{2}}, \end{array}$$

where *a*, *b*, and *c* are arbitrary real numbers. The Gaussian curve graph is a characteristically symmetrical “bell curve” shape, where *a* represents the height of the peak of the curve, *b* is the position of the center of the peak, and *c* is called the standard variance, which is a parameter used to control the width of the “bell.” Let *a* = 1, *b* = *μ* (mean value) and *c* = *σ* (standard variance); the Gaussian distribution can be obtained as follows:

(2) $$\begin{array}{c} G\left(x\right)=e^{-{\left(x-\mu \right)}^{2}/2\sigma^{2}}. \end{array}$$

Its function curve is shown in Figure 3.

The horizontal axis represents the possible values, the vertical axis represents the probability distribution density *G*(*x*), the expected value *μ* of the normal distribution determines the center of the curve, and the standard variance *σ* determines the magnitude of the distribution. In Figure 3, the settings are *a* = 1, *b* = *μ* = 0. Hence, the peak heights and center positions of all curves are the same. With increasing standard variance, the graph becomes wider, the distribution becomes dispersed, and the area of the graph becomes increasingly larger. The closer the value of *x* is to the center, the greater the value of *G*(*x*). Therefore, we can use this feature of the Gaussian function by assigning the distance from the pixel's location to the center point of the patch as the input *x* to the Gaussian function and calculating the weight coefficient of each pixel point through Gaussian function [11].

### 3.2. The Proposed Patch Fusion Method

In Figure 4, the blue part is patch 1, *B* is the central point of patch 1, the orange part is patch 2, *C* is the central point of patch 2, and the red part is the overlapping part of these two patches. It can be seen that pixel *A* is closer to the central point *B* in patch 1 in the overlapping area, so its predicted value in patch 1 is more accurate. To reduce the weight of the predicted value of the pixel located at the boundary, we convert the Euclidean distance between the pixel and the center of the patch to the weight coefficient of the pixel through the Gaussian truncation function. The formula is defined as follows [11, 12]:

(3) $$\begin{array}{c} W\left(y\right)=\left\{\begin{array}{c} \frac{1}{z}e^{-{\left|y\right|}^{2}/2\sigma^{2}},\;\text{for }\left|y\right|\leq \rho ,\\ 0,\;\text{else}, \end{array}\right. \end{array}$$

where *σ* represents the standard variance, *z* represents the normalization factor of the normalized Gaussian kernel, and *ρ* represents the radius to measure the size of the local region. Therefore, in Figure 4, assuming that the predicted value of point *A* in patch 1 is *P*_*AB*_ and the predicted value in patch 2 is *P*_*AC*_, the final predicted value of point *A* is *P*_*A*_ = *W*(*y*1)*P*_*AB*_ + *W*(*y*2)*P*_*AC*_.

We take a two-dimensional graph as an example. Assuming that the image size is *M* × *N*, the patch size is *h* × *w*, and the stride size is *s*, *n* patches can be generated, and the value of *n* can be calculated by

(4) $$\begin{array}{c} n=\left\lfloor \frac{M-\left(h-s\right)}{s}\right\rfloor \left\lfloor \frac{N-\left(w-s\right)}{s}\right\rfloor . \end{array}$$

In these *n* patches, the Gaussian distribution of the distance between each pixel point and the center point of the patch is the same, which is calculated by Formula (2). The Gaussian function value corresponding to the pixel point (*i*, *j*) in the *k*th patch can be recorded as *G*_*k*_^(*i*, *j*)^(*y*_*k*_), *k* ∈ [1, *n*], where *y*_*k*_ is the Euclidean distance from this point to the central point of the patch. Therefore, Formula (3) can be expressed by *G*_*k*_^(*i*, *j*)^(*y*_*k*_).

(5) $$\begin{array}{c} W\left(y_{k}\right)=\left\{\begin{array}{c} \frac{1}{z}G_{k}^{\left(i,j\right)}\left(y_{k}\right),\;\text{for }\left|y_{k}\right|\leq \rho ,\\ 0,\;\text{else}, \end{array}\right. \end{array}$$

(6) $$\begin{array}{c} m_{i}=\left\{\begin{array}{c} \left\lfloor \frac{i}{s}\right\rfloor +1,\;i<h,\\ \frac{h}{s},\;h\leq i\leq \left\lfloor \frac{M-\left(h-s\right)}{s}\right\rfloor s-1,\\ \left\lceil \frac{\left(\left\lfloor \left(M+s\right)/s\right\rfloor -1\right)s-i}{s}\right\rceil ,\;\left\lfloor \frac{M-\left(h-s\right)}{s}\right\rfloor s-1<i<\left(\left\lfloor \frac{M+s}{s}\right\rfloor -1\right)s,\\ 0,\;\left(\left\lfloor \frac{M+s}{s}\right\rfloor -1\right)s\leq i. \end{array}\right. \end{array}$$

Assuming that the pixel point *O*(*i*, *j*) overlaps *m* times, *m* = *m*_*i*_ × *m*_*j*_,  *i* ∈ [0, *M* − 1], *j* ∈ [0, *N* − 1], then *m*_*i*_ can be calculated by Formula (6) [9], and the edge part that cannot be obtained by the patch is discarded. The value of *m*_*j*_ can be obtained by replacing *M* in Formula (6) with *N*. Assuming that the *m* predicted values of the pixel point are *P*^(*i*, *j*)^ = {*p*_1_^(*i*, *j*)^, *p*_2_^(*i*, *j*)^, ⋯, *p*_*m*_^(*i*, *j*)^} and the weight coefficients of the *m* predicted values calculated by Formula (5) are *W*^(*i*, *j*)^ = {*W*_*y*1_^(*i*, *j*)^, *W*_*y*2_^(*i*, *j*)^, ⋯, *W*_*ym*_^(*i*, *j*)^}, then the final predicted value of the pixel point *O*(*i*, *j*) is

(7) $$\begin{array}{c} {\overset{\wedge }{P}}^{\left(i,j\right)}=P^{\left(i,j\right)}\cdot W^{\left(i,j\right)}=\overset{m}{\underset{k=1}{\sum }}p_{k}^{\left(i,j\right)}W_{y_{k}}^{\left(i,j\right)}, \end{array}$$

where ∑_*k*=1_^*m*^*W*_*y*_*k*__^(*i*, *j*)^ = 1.

## 4. Experimental Results and Analysis

To evaluate the effective fusion ability of the algorithm, we employed DN-RESnet (a deep convolutional neural network consisting of several residual blocks) [13] as the training model. The bias field removal experiment was carried out on the simulation database BrainWeb [14–15] and the real dataset HCP (Human Connectome Project) [16]. Meanwhile, we also used the DnCNN (De-nosing Convolutional Neural Network) denoising model [17] for validation on the IXI-Guys (http://brain-development.org/ixidataset) dataset [18].

### 4.1. Validation of the Proposed Fusion Method in the Bias Removal Model

#### 4.1.1. Results Obtained on the Simulation Database BrainWeb

In the Simulated Brain Database (SBD) [15], the size of each MRI brain image volume is 181 × 217 × 181 voxels with a resolution of 1 × 1 × 1 mm3. 2D MRI slices were extracted from the volumes for training and testing, with different intensity nonuniformity (INU) levels (20%, 40%, and 60%) on the axial plane, respectively. We used rotation, mirror imaging, translation, and other methods to expand the samples. Finally, 604 slices were obtained for training and 30 slices for testing from the volume of each INU level. In order to obtain fewer redundant regions, we cropped the edges of each slice, so the slice size becomes 210 × 180. In the training stage, we set the patch size to 60 × 60, and obtained 99 patches from each image by using a sliding window with a stride of 15 × 15. Finally, we obtained 59796 patches.

In our algorithm, we needed to set the value of the standard variance*σ*. We conducted experiments on datasets with different (INU) levels (20%, 40%, and 60%) setting the value of *σ* in the range of 1 to 20. The mean square error (MSE) and the structural similarity index (SSIM) were used as the quantitative evaluation criteria after image reconstruction. The results are shown in Figures 5 and 6.

It can be seen from Figures 5 and 6 that when the INU level is not high (20%, 40%), no matter what the value of the standard variance *σ* was, it had little effect on the MSE and SSIM after image reconstruction. However, when the INU level increased to 60%, MSE and SSIM values fluctuated for different values of *σ*. When *σ* = 4, MSE and SSIM showed better performance. At the same time, we also performed the same experiments on the real dataset HCP [16] and reached at consistent conclusions. Therefore, in the bias removal experiment of our algorithm, the standard variance *σ* was set to 4.

To evaluate the fusion ability of the proposed method after image reconstruction, we compared the proposed method with popularly available and state-of-the-art nonoverlapping patch splicing (NPS) method, arithmetic average weighted method (AAW) [5], MIScnn [7], Pathify [8], and Exponential-Distance-Weighted method (EDW) [9] on three datasets with different INU levels from BrainWeb. The dataset with INU = 20%and noise level = 3% was denoted as n3-20, the dataset with INU = 40%and noise level = 0% was denoted as n0-40, and the dataset with INU = 60%and noise level = 0% was denoted as n0-60. The experimental results are shown in Figure 7, Table 1, and Figure 8.

In Figure 7, we show the bias field images fused by different methods. The bias field images of NPS (Figure 7(c)) and Pathify (Figure 7(f)) demonstrate an obvious blocking artifact phenomenon, while the blocking artifact phenomena of AAW (Figure 7(d)) and MIScnn (Figure 7(e)) are greatly improved, but the seam line between patches are vaguely visible. The AAW method is greatly affected by the stride. The larger the stride is, the more obvious the blocking artifact phenomenon is. However, in Figure 7(e), the MIScnn method also shows the phenomenon of uneven bias field, indicating the inaccurate prediction of the edge region. EDW (Figure 7(g)) and our method (Figure 7(h)) consider the uncertainty of edges and assign different weights to the central region and the edge region, effectively eliminating the grid artifacts. From Table 1 and Figure 8, it is observed that on the n0-40 dataset, our method has little difference from the EDW method, but on the n3-20 and n3-60 datasets, our method shows better performance in the quantitative evaluation of MSE and SSIM than EDW, indicating that our method has better generalization ability.

#### 4.1.2. The Results from the Real Database HCP

HCP [16] real human brain dataset contains T1-W and T2-W structural MR images of healthy adults from Siemens Skyra 3T scanner, along with the corresponding bias fields images. For detailed information, please refer to [19]. In the experiment, we randomly selected the T1-W structural images of 10 patients from the dataset. The size of each MRI brain image was 260 × 311 × 260 voxels, and the resolution was 0.7 × 0.7 × 0.7 mm^3^. We randomly selected 1000 slices from these 10 brain image volumes. To better train the model, we augmented the data with rotation and mirroring methods and finally obtained 3200 training samples and 200 testing samples. Similarly, to speed up the training process and obtain fewer redundant regions, we cropped the image edges of each sample with size 300 × 240. In the training stage, we set the patch size to 60 × 60 and obtained 63 patches from each image by using a sliding window with a stride of 30 × 30. Finally, we obtained 201600 patches.

In Figure 9, we show the bias field images from HCP fused by different methods and the corrected images. It can be seen that the bias field images fused by the NPS, AAW, MIScnn, and Pathify methods have obvious seam lines at the junction between patches, which indicates that the prediction at the boundary region is not accurate. EDW and our proposed method can effectively reduce grid artifacts by assigning different weights to pixels in different regions. In the enlarged red box of the corrected image, it can be seen that there are no grid artifacts in Figures 9(g) and 9(h). Meanwhile, it can be seen from Figures 9(g) and 9(h) that the bias field obtained by our method is smoother, and the intensity of each tissue area of the corrected image looks more consistent, which is obvious in the white matter region of Figure 9(h). This conclusion is also verified in Table 2. Our method can obtain a lower MSE value and a higher SSIM value.

In the AAW method, the stride size has a great influence on the patch fusion effect. Therefore, on the HCP dataset, we verified the effect of different stride sizes on the fusion effect of AAW [5], EDW [9], and the method proposed in this paper.  Table 3 lists the number of patches obtained on each image with different stride sizes and the fusion time of these three methods. At the training stage, we used a sliding window with a stride of 30 × 30 to obtain 63 patches from each image and finally obtained 201,600 patches. At the test phase, according to Equation (6), we used sliding windows of different strides to extract patches as shown in Table 3 and explored the performance of the proposed fusion method.

In Figure 10, we can see that the AAW method (Figure 10(b)) is greatly affected by the stride size. When the stride size is 10 × 10, the image blocking artifact is not obvious in the fused bias field image, but with increasing stride size, obvious grid artifacts appear in the fused image. The EDW method (Figure 10(c)) and our method (Figure 10(d)) are less affected by the stride size. From the line chart of the quantitative evaluation index MSE in Figure 11, we can see that the highest point of the AAW method fluctuates by approximately 9% relative to the lowest point, while the highest point of the EDW method and our method fluctuates by less than 1% relative to the lowest point %. In Figure 12, we show the change in SSIM value with the change in stride size. The SSIM value of the AAW method decreases obviously with increasing stride. Although the SSIM values of the EDW method and our method fluctuate with the change in stride, their amplitude is small. In addition, compared with the EDW method, our method resulted in a smoother bias field image. As seen from Figure 12, our method can obtain a higher SSIM value than the EDW method despite the INU level, regardless of stride size.

As seen in Table 3, the smaller the step size, the more the number of patches extracted from each image; hence, the fusion time increases accordingly. Although the AAW method can obtain a relatively smooth bias field image when the stride is 10 × 10, the fusion time difference is very small compared with the other two methods when the stride is 30 × 30. However, there are still blocking artifacts in the images fused by the AAW method. Our method and the EDW method are less affected by the stride. Even when the stride is 30 × 30, the bias field image obtained does not appear to contain image blocking artifacts, having a lower MES value and higher SSIM value than the AAW method. Therefore, in the experiment on HCP database, to shorten the fusion time, we uniformly used a sliding window with a stride of 30 × 30 to extract patches.

### 4.2. Validation of the Proposed Fusion Method on the Denoising Model for 3D Brain MR Images

To further evaluate the fusion performance of the proposed algorithm, we adopted the DnCNN denoising model [18] for validation on the IXI-Guys human dataset. We randomly selected 20 T1w brain images from the IXI-Guys dataset with an image size of 256 × 256 × 150 and voxel resolution of 0.9375 × 0.9375 × 1.2 mm^3^ [20, 21]. 12 images were randomly selected as the training set, 4 images were used for verification, and the other 4 images were used for testing. In this dataset, we manually added 30% Rician noise to simulate the noise image [22]. In order to better train the model, we cropped the image to 240 × 240 × 150, used the mirroring method to augment the data, and finally obtained 36 training samples. For patch-based training, we set the patch size to 60 × 60 × 60 and used a sliding window with stride 30 × 30 × 30 to obtain 196 patches from each image. Finally, we obtained 7056 patches for training the 3D model. Our fusion algorithm is evaluated on the testing set based on three aspects: MSE, PSNR (peak signal-to-noise ratio), and SSIM. The results are shown in Table 4.

In Table 4, we quantitatively compared the image qualities of the proposed fusion method and the state-of-the-art fusion methods in terms of MSE, PSNR, and SSIM [23] by training the denoising model on the 3D IXI-Guys human dataset. As seen from Table 4, the fusion method proposed in this paper shows lower MSE and higher PSNR and SSIM than other methods, which further proves the effectiveness of our method. In addition, in the enlarged red box in Figure 13, it can be seen that the denoising images of NPS, AAW, MIScnn, and Pathify have obvious seam lines between patches, which further illustrates the difference in the prediction of boundary regions between adjacent patches. However, in Figures 13(g) and 13(h), this situation is much better, because both the EDW method and our method fully consider the uncertainty of the edge and assign different weights to the central and the edge regions to solve the problem. However, a small grid artifact appears faintly in Figure 13(g), while in Figure 13(h) obtained by our fusion method, there is no grid artifact and is smoother than EDW.

## 5. Discussion and Conclusions

In deep learning, when the resolution of the image to be processed is too large and the resources (such as video card and video memory) are limited, the image is divided into small patches for processing, and the image patches are reconstructed and then spliced. Since the zero-padding method is commonly used in deep learning networks to ensure the consistency of input and output sizes, this method can lead to uncertainty in edge prediction. After image reconstruction, obvious blocking artifacts appear in the spliced image due to the inconsistency of the boundary information of each patch processed. To solve this problem, we have studied the most popularly available patch fusion methods and proposed a fusion method with a truncated Gaussian function as a weighting function to assign weights to each pixel in the patch. In this method, we used the weighting function to convert the Euclidean-distance between the overlapping point and the central point of the patch into a weight coefficient, considered the predicted pixel values in all patches, and reduced the weight of the predicted pixels at the boundary. Finally, we obtained the predicted pixel values through the weighted calculations.

We carried out experiments on the simulated database BrainWeb and the real dataset HCP using the bias removal model. After comparing the proposed method with the popularly available fusion methods, NPS, AAW, MIScnn, patchify, and EDW, our method can obtain a super seamless and smooth bias field image. As evidenced by quantitative analysis, our fusion method achieves lower MSE and greater SSIM on both simulated and real data, which is clearly superior to the other five methods. In addition, we also discussed the bias field images obtained by AAW, EDW, and our proposed method with different stride on the HCP dataset. To further demonstrate the robustness of our method, we conducted experiments by training a denoising model on the IXI-Guys human dataset. Experimental results show that our fusion method also performs better than other five methods in quantitative analysis of MSE, PSNR, and SSIM on 3D dataset. However, our method has two shortcomings: (1) the standard variance of Gaussian function *σ* needs to be determined. Different application backgrounds require different values of *σ*. For example, in the bias removal model, the best fusion performance is achieved when *σ* = 4, while on the 3D brain image denoising model, the best fusion performance is achieved when the value of *σ* is around 8; (2) while our approach for obtaining an artifact-free image under a wider sliding window takes about the same amount of time as the AAW method for obtaining the same quality image under a smaller stride, it still takes a lengthy period. In a future work, we hope to be able to adaptively select the hyperparameters of different scenes and further optimize the algorithm to shorten the running time.

In this paper, we introduced a truncated Gaussian function as a weighting function, which converted the Euclidean distance between each pixel in the patch and the center point into the weight coefficient of this pixel, to reduce the image blocking artifact in patch-based image reconstruction. We demonstrated that the method proposed in this paper has significant advantages over existing patch fusion methods. Additionally, our approach can be applied to any patch-based deep learning model, even when the model is already trained.

## Figures and Tables

**Figure 1:** Image blocking artifacts after patch-based image reconstruction.

**Figure 2:** Three methods for extracting patches of images.

**Figure 3:** The Gaussian function curve (*a* = 1, *b* = *μ*, *c* = *σ*).

**Figure 4:** Schematic diagram of patch overlap. The red part is the overlapping area, and *B* and *C* are the center points of patch 1 and patch 2, respectively. *A* is a point in the overlapping area, and *y*1 and *y*2 are the distances from point *A* to the two center points.

**Figure 5:** MSE values of different standard variance on different INU level datasets.

**Figure 6:** SSIM values of different standard variance on different INU level datasets.

**Figure 7:** Contaminated image, real image, and bias field images obtained by different fusion methods from the BrainWeb database: (a) original image (INU = 40%, noise level = 0%); (b) real image; (c) NPS; (d) AAW; (e) MIScnn; (f) pathify; (g) EDW; (h) proposed method.

**Figure 8:** SSIM values between the real image and the corrected images obtained by different fusion methods.

**Figure 9:** Bias field images obtained by different fusion methods on real HCP data and corresponding corrected images: (a) original image, (b) real image, (c) NPS, (d) AAW, (e) MIScnn, (f) pathify, (g) EDW, and (h) proposed method.

**Figure 10:** Bias field images obtained by fusing patches with AAW, EDW, and the proposed methods under different strides. (a) The original image and the real image. (b) The result of AAW. (c) The result of EDW. (d) The result of the proposed method. The step sizes from left to right are 10 × 10, 20 × 20, 30 × 30.

**Figure 11:** MSE values of AAW, EDW, and the proposed methods using different strides on the HCP dataset.

**Figure 12:** SSIM values of AAW, EDW, and the proposed methods using different strides on the HCP dataset.

**Figure 13:** Images from the IXI-Guys dataset with 30% level Rician noise, real images, and denoised images obtained by different fusion methods: (a) noise image, (b) noise-free image, (c) NPS, (d) AAW, (e) MIScnn, (f) pathify, (g) EDW, and (h) proposed method.

**Table 1:** MSE values between the real image and the corrected images obtained by different fusion methods.

Methods	n3-20	n0-40	n0-60
NPS	13.60 × 10^−4^	2.139 × 10^−4^	8.228 × 10^−4^
AAW [5]	16.95 × 10^−4^	2.054 × 10^−4^	6.575 × 10^−4^
MIScnn [7]	48.57 × 10^−4^	2.108 × 10^−4^	7.079 × 10^−4^
Pathify [8]	13.53 × 10^−4^	2.110 × 10^−4^	7.985 × 10^−4^
EDW [9]	6.593 × 10^−4^	2.053 × 10^−4^	7.887 × 10^−4^
Proposed	4.193 × 10^−4^	2.051 × 10^−4^	6.212 × 10^−4^

**Table 2:** The MSE values, SSIM values and synthesis time between the real image and the corrected image obtained by different fusion methods.

Method	NPS	AAW [5]	MIScnn [7]	Pathify [8]	EDW [9]	Proposed
MSE	1.233∗10^−3^	1.130∗10^−3^	1.136∗10^−3^	1.468∗10^−3^	1.139∗10^−3^	1.104∗10^−3^
SSIM	0.9882	0.9909	0.9913	0.9869	0.9936	0.9942
Time (s)	0.25	0.40	0.41	0.39	1.79	1.81

**Table 3:** The number of patches extracted from each image with different strides and the fusion time.

Stride	10 × 10			20 × 20			30 × 30		
Patch number	475			130			63		
Fusion time (s)	AAW	EDW	Proposed	AAW	EDW	Proposed	AAW	EDW	Proposed
	1.77	6.16	6.20	0.61	2.44	2.45	0.37	1.79	1.81

**Table 4:** Average MSEs, PSNRs, and SSIMs of different fusion methods on the IXI-Guys dataset.

Method	NPS	AAW [5]	MIScnn [7]	Pathify [8]	EDW [9]	Proposed
MSE	4.574∗10^−4^	3.034∗10^−4^	3.024∗10^−4^	3.064∗10^−4^	2.986∗10^−4^	2.971∗10^−4^
PSNR	32.85	35.64	35.67	35.61	35.71	35.76
SSIM	0.9789	0.9833	0.9838	0.9835	0.9841	0.9843

## Data Availability

All datasets used in this study are discussed in Section 4. They are publicly available and cited in the list of references.
